# Cleanup Sketched Drawings: Deep Learning-Based Model

This article has been retracted.

**DOI:** 10.1155/2022/2238077

**Published:** 2022-05-06

**Authors:** Amal Ahmed Hasan Mohammed, Jiazhou Chen

**Affiliations:** College of Computer Science and Technology, Zhejiang University of Technology, Hangzhou, China

## Abstract

Rough drawings provide artists with a simple and efficient way to express shapes and ideas. Artists frequently use sketches to highlight their envisioned curves, using several groups' raw strokes. These rough sketches need enhancement to remove some subtle impurities and completely simplify curves over the sketched images. This research paper proposes using a fully convolutional network (FCNN) model to simplify rough raster drawings using deep learning. As input, the FCNN takes a sketch image of any size and automatically generates a high-quality simplified sketch image as output. Our model intuitively addresses the shortcomings in the rough sketch image, such as noises and unwanted background, as well as the low resolution of the rough sketch image. The FCNN model is trained by three raster image datasets, which are publicly available online. This paper demonstrates the efficiency and effectiveness of using deep learning in cleaning and improving the roughly drawn image in an automatic way. For evaluating the results, the mean squared error (MSE) metric was used. From experimental results, it was observed that an enhanced FCNN model reported better accuracy, reducing the prediction error by 0.08 percent for simplifying the rough sketch compared to the existing methods.

## 1. Introduction

Drawing is one of the artistic intellectual skills that allow ideas to be transformed into artistic images. Drawn either on paper with a crayon or on a tablet with a digital pen, line drawings are used in certain cases, such as drawing or showing the contours or shapes of objects. The priority is to rapidly express concepts and ideas instead of showing fine details, which leads to coarse and rough line drawings. The design is refined based on input from an initial sketch until the final element is created. This recurrent refining requires artists to constantly clean up and simplify their raw drawings, which significantly increases their burden. It is very time-consuming and tedious to trace the rough drawing by hand for a clean drawing. There are two types of processes for rough image cleanup: simplification and vectorization.

Vector graphics are a lightweight digital graphic format that uses primitive mathematical material to represent lines and curves. Vector graphics can be rasterized optimally concerning the basic resolution in analytical procedures. Because parameters and control points can be altered programmatically or through user interfaces, vector graphics are versatile and simple to utilize. Vector graphics, as opposed to raster images, can be altered without affecting the quality of the image. As a result, vector graphics are now used in various technical content production workflows, such as computer-supported design, UI design, and 2D animation. The vectorization of line drawings is to convert a bitmap into a vector graph (vector graphics comprise many geometrical shapes such as lines, dots, curves, and multigroups). Through the modeling of graphical elements with parametric curves, such as Bézier splines [1], vector graphics have many advantages over bitmaps. Such automatic vectorization work seems to be acceptable in our eyes, but it presents major computing challenges. Simplifying the image's editing and repurposing by scanning or filming it would make it an important research topic in computer animation and image processing. After eliminating noise influences, preserving the topological structure of the original line drawing during the simplification process is the hardest thing to do [2, 3].

A pixel-wide stroke skeleton was generated from input drawings using traditional vectorization methods [4–7] before vector curves were fitted into those branches. As a result, they were the best-adapted methods for vectorizing “clean” or simplifying sketch images, where strokes with the same envisioned curves clustered partially or completely. Stroke skeleton branches for dangling strokes of sketch images were obtained through morphological thinning by Noris et al. [7] and Bartolo et al. [8]. Favreau et al. [9] have combined two vertices of skeleton branches at valence and collapsed short branches by the operations of simplifying and vectorizing the skeleton of the image. Additionally, these operations have functioned effectively to improve the overall accuracy that equalizes a simple process with input fidelity. Aside from that, optimization did not affect more difficult operations, such as joining corresponding branches of sketch images. Simplification methods used by Noris et al., Favreau et al., and Hilaire et al. [6, 7, 9] concentrated on curve network topology abstraction and cleaning up. Lately, Bessmeltsev et al. [10] developed a sketch vectorization process. They used a polyvector method to direct the positioning of primitives. Their proposed method used an advanced range of adjustable heuristics for building curve networks and cleaning up topology, which was difficult to modify and yielded clean vectorization of technical designs with low primitives.

To simplify raster drawings, deep learning techniques facilitated the process of improving and cleaning the rough sketches. Simo-Serra et al. [11] introduced a convolutional neural network-based model to decrease MSE loss. However, the loss of MSE usually results in a blurring of the clean line drawing. To deal with the problem of blurring, Simo-Serra et al. [12] sproposed generative adversarial networks (GANs), which integrate adversary loss into the loss function. Since GAN assures only local cleanliness while less attention is being paid to the overall semantic structure, this method can solve blurring but cannot yet handle immensely sketchy strokes. Such methods face the challenge of working on raster sketches. The rough sketch drawings suffer from some defects, including the extra lines and the gaps in distance between the intersections of the strokes. Sometimes, the grey colors in the background need to be removed. The noise in rough sketches ruins the beauty of the sketch image. Nonetheless, even though the information in our input bitmaps is smaller than that in digital strokes, our technique delivers high-quality results when applied to rasterized drawings.

This paper proposes an automatic approach to convert rough sketch images into simplified clean drawings. This approach overcomes the complexity of the mathematical operations of vectorization. The advantage of our proposed approach is that it accepts rough sketch images of any size as input and yields high-quality simplified sketch images as output automatically. The result of our approach is a cleanup of sketching images from some impurities that misrepresent the beauty of the image. By deleting any unexpected regions and open curves while retaining the drawing structure desired by the user, Figure 1 shows a sample of the rough sketch image as input and the rough cleanup sketch image as the result after it is cleaned up by our model. The model is trained on raster sketch datasets, which are collected from some publicly available sources on the internet. The dataset images are made up of two parts. The first part consists of rough sketch images, and the second part is manually enhanced and cleaned up images. With the help of image enhancement software such as Photoshop, these two parts are cleaned and enhanced by experts in the field of graphic art.

To ensure that our strategy is effective, we compare it to other approaches by performance measurements such as model training accuracy, model loss, and time complexity. Compared with state-of-the-art methods, our method with the availability of deep learning techniques outperforms them with high accuracy.

## 2. Related Work

In this section, we reviewed some previous studies related to sketch image cleaning and enhancement. Based on the techniques used, this section divides the simplification and vectorization methods into two subsections: nonlearning-based (field-based, fitting-based) ones and learning-based ones.

### 2.1. Non-learning-Based Methods

#### 2.1.1. Field-Based Approaches

For field-based approaches, a wide range of algorithms have been published for vectorizing line drawings. Rough sketches consist of several, almost parallel strokes. This discovery prompts scientists to filter certain drawings with anisotropic blurring kernels [7–9]. A public concept of such methods is the orientation of the blurring kernels to the strokes according to a vector field. However, at connections, where several leading directions occur, tangent vector fields become unspecified. Frame fields [13] provide a way to address this challenge by representing at every point of the drawing two dominant directions that allow the exact capture of *T*- and *X*-junctions. The field's singularities can also capture high-valence junctions. Various recent approaches have taken advantage of the setting field demonstration for sketch processing by Bessmeltsev and Solomon [10] on line drawing vectorization. In addition to the approaches for sketch-based models by Iarussi et al. [14] and Li et al. [15].

To vectorize freeform lines, the tracking methods measure first the image's tangential field and then trace streamlines with integral line convolution. A variety of current methods are found for direction field estimation. The central line streamlines Bao et al. [4] traced directly from the seed point at the centre of the line or Nieuwenhuizen et al. [16] as the midpoints of two contour streamlines that start from seed points at the boundary line. Special corrector mechanisms must be used for both cases to evade gathering faults in the tracing development, for example, the Kalman filter from Bartolo et al. [17], 2D square fitting, and the Runge-Kutta algorithm [18]. And Bao and Fu have proposed a trace-based vectorizing system that uses cross-sections to accurately trace lines of almost constant width [4]. They drew precise tracing directions centered on a field of orientation and smoothness automatically to evaluate and presuppose nearly constant line width. The whole vectorization took a few seconds to complete. Their methodology collected far more details than Illustrator. The resulting lines were visually pleasing in their entirety. However, not all the data is guaranteed to be extracted, especially in small ambiguous regions. And due to the antialiasing effect, each line is perhaps vaguer in its entries.

An increasing amount of literature on vectorizing line drawings has been published in recent years. Modern algorithms also cannot reveal junctions or locations where the curves intersect even if they are clean lines; this results in vector drawings with incorrect connectivity. Bessmeltsev et al. [10] offered a vectorization method based on cutting-edge mathematical algorithms for frame-field processing. As part of an approach presented by Chen et al. [18], it has been used for sketch image vectorization with a global variation approach for junction disambiguation. They use tangent fields, as shown in Figure 2, which cannot catch a group of directions at a sketch's junction point. The Chen et al. approach [18] relied on user interaction and arbitrary thresholds for the resolving junctions. Their approach did not even take account of the topology of the drawing, which can give rise to disconnected lines or fake connections. On that basis, Bessmeltsev et al.'s approach employed a more natural representation to track the junctions in drawings. The two directions in the frame field were disambiguated around the *T*- or *X*-junctions, and their varied nature resisted noise. However, they did not support shady regions, and rough sketches with multiple overlaps may require more simplification, while very low-resolution images are difficult to vectorize.

To extract vector curved networks, Stanko et al. [19] proved that their approach effectively vectorizes both the clean and rough lines of drawings, whereas previous methods were based solely on one form of drawing. A strength of their method is their ability to combine parallel strokes by increasing the grid parameterization scale, but the production of complex sketches took several minutes. Their global solution needs parameterization for the whole mesh, even though the adjustments are localized to specific regions in the drawing when the user updates the mask. Also, their frame field regularization strategy can struggle around very sharp intersections, leading to a locally incorrect topology. Because its parameterization cannot bifurcate an isoline, these field configurations lead to local parametric inversions; the resulting isolines, in practice, “loopback” on their own until they enter a mesh boundary. Using their vertex frame region, high-valence junctions can be hard to catch.

#### 2.1.2. Fitting-Based Approaches

Fitting-based methods are used for the identification of more complex primitives such as ellipses [20] and Bezier curves [1]. They are therefore still limited to particular primitives; so, free-form line designs cannot be recognized. A considerable amount of literature was published on this issue; Hilaire and Tombre [6] introduced a system to vectorize the graphic sections of paper line drawings. To accomplish this, the binary image input is divided into layers of uniform thickness, each layer is skeletonized, random sampling is performed, and the results are simplified, but the technique is currently limited to identifying straight segments and circular arcs, but can be generalized to other primitives. Being a noncontextual process, some situations (for example, *X* junctions with tiny opening points) where clear contextual information rules could possibly lead to accurate and correct graphical interpretations also fail.

Pham et al. [21] implemented a junction identification and characterization method in line drawing pictures. As this method worked with line-like primitives, its output would degrade as it was extended to fill objects like logo images. Furthermore, the process of junction optimization may lead to problems in interpreting the junction location incorrectly as that created by the craftsmen. However, this argument is accurate in some areas of precise line drawing, like vectorization, but it is also interesting to detect local features to deal with the problems of large-scale document indexing and retrieval. The low incidence of false positives is not problematic for the final findings in this sense. The observed joints should also be used along with other types of characteristics (e.g., endpoints, isolated straight lines, arches, and circles) for the full representation of document pictures. Favreau et al. [9] introduced the first vectorization algorithm that specifically combines input bitmap fidelity and output simplicity, calculated by the number and grade of curves. They also illustrated the robustness of their algorithm in a range of sketches, drawings, and raw scheme drawings. Their algorithm was not intended to handle missing data, such as broken strokes. Their algorithm provides a relationship between simplicity and accuracy, which is controlled by the as expressed in Equation (1) [9]. However, their algorithm did not take into account strong geometric regularities, such as parallelism, orthogonality, or symmetry. In clean drawings consisting of small areas, it sometimes excluded fine details and did not extract open curves. It is weak in the presence of gaps. Most of the work previously done cannot extract a simplified topology for drawings consisting of several unnecessary lines.

(1) $$\begin{array}{c} \text{U}\left(x\right)=\left(1-\lambda \right)\text{Ufidelity}\left(x\right)+\mathrm{\lambda Usimplicity}\left(x\right). \end{array}$$

In 2018, Chen et al. [22] showed that their enhanced topology benefits their vectorization system and present topology-driven methods and helped them robustly and efficiently vectorize rough drawings. The trapped-ball algorithm they used is not susceptible to small gaps between the neighboring areas and cannot connect large gaps. And when they are closed, it is also difficult to distinguish strokes because the trapped-ball algorithm appears to combine them. In certain special cases, their assumptions about the area and open curve elimination priority have also been violated. When making sketches for lines, artists often represent envisioned curves by utilizing several closely grouped or overspent strokes. Assuming that drawings are accurate, human viewers can easily perceive the planned, combined, and curved mental images of the artist. Stroke aggregator [23] considerably improved the state of the art and created cumulative curve drawings that are confirmed in line with the expectations of the audience. They can benefit from a variety of design and sketch-based modeling systems intended to function with associated expected curve fitting. The fitting step aims to match a polyline curve to a polyline stroke group. When calculating the curve, they tried to capture the intended form of the artist and specifically maintained the slopes or tangents of the strokes. An updated moving least squares (MLS) algorithm was used to calculate the optimal curve [24, 25]. The standard MLS formulation did not help tangent optimization, as the tangent treatment required information on points of order that was not available in the MLS setting. Alternatively to MLS optimization, the construction of a nonoriented gradient field by Chen et al. [26] may provide tangential information; however, the resulting tangents also need a clear focus. Their method helped to resolve ambiguities in the data. However, their approach was based on the native stroke setting only. It can fail, therefore, in circumstances in which stroke levels are unreliable. Strokes were used in the sketches as expressive paint brushes, and their tangents no longer represented the tangent of the matching collective curves. In this case, the principal indicators of angular compatibility among cluster strokes are miscarried.

In 2019, Liu et al. [27] suggested a technique for vector sketch simplification based on a detail of the geometric construction, which is called base complex mining from the input vector grid. Their algorithm is applied to arbitrary vector graphs. The patch-patch fusion was achieved via easily merging two patches with a similar edge into another. These patches extend unseeingly, which can be devoid of decreasing and lead to the emergence of borderlines between the patches. This phenomenon is particularly obvious if a substantially irregular graph is used. Boundary patches can be fixed through the postprocessing step, that can be done by reassembling the curve. The effects of reassembling simplification are not desired if the boundary patches are significantly broad.

Recently, PolyFit was proposed by Dominici et al. [28]. It is a vectorization technique that produces well-matched vectorizations with human preferences. It is particularly suitable for inputs with low resolution. The proposed method calculates a polygonal fit by expending a dynamism function based on perception and using its output as an input to a trained classifying unit. However, they only made a mistake on nine inputs, citing cases where users preferred the unconventional result over either theirs or both. Their implementation only regulated individual borders, and their procedure is susceptible to minor raster changes and regularity imperfections such as symmetries.

### 2.2. Learning-Based Methods

Lately, deep learning has been validated as an efficient method that is aimed at simplifying sketches on a raster basis. Current approaches require vector images to simplify drawing as an input. Simo-Serra et al. (2016) [11] permitted more overall and demanding feedback of rough raster sketches like those produced from pencil screens. It depended heavily on the quality and amount of the training data. However, they showed that even with a small dataset, several different images can still be generalized very well. Furthermore, even if the model implications are very fast, the learning task is computer-priced and relies on high-end GPUs for a reasonable amount of time to complete.

Sasaki et al. [2] proposed identifying and completing gaps in alignment drawings by the convolutional neural network automatically. However, their method was confused by very multifaceted structures and did not perform better when employing the mask; very large regions that were missing were also difficult and could fail to fill the gap properly. It also purified the nongap lines and contrasts strongly with state-of-the-art approaches that required masks as input. At the beginning of 2018, Simo-Serra et al. [12] transformed difficult rough drawings into clean line drawings and suggested a simplification approach that can outperform current approaches. In addition, its proposed structure can also be used to deal with the inverse problem. While its approach can make effective use of unregulated data, it still relies heavily on supervised quality data, which could not achieve good results (in general, the absence of managed supervision did not tolerate maintaining fine details). The model found it difficult to eliminate shading from the input image instead of retaining the unwanted output lines.

Ha and Eck [29] developed a method to model drawings with recurring neural networks. They have generated clear drawings using a vectoring format and made the training more robust. The proposed method could provide a way to complete unfinished drawings and code existing sketches into a latent vector and create identical, latent space designs. However, the sketch based on the RNN technique was skilled at modeling sketches up to 300 data points. The model becomes steadily more difficult to train on the far side of this length. For more complex image types, such as mermaids or lobsters, the metrics for reconstruction loss were not as strong as for simple sketch images like ants, faces, or fire trucks. Also, sketch RNN was ineffective in simultaneously modeling a large number of classes. Incoherent samples were generated from the model's classes, with discrete sketches displaying attributes from multiple classes. In 2019, photosketching [30] achieved state-of-the-art success in the identification of outstretched boundaries, indicating that contour drawing can be a simpler and more interesting alternative to boundary note drawing. However, boundary detection on its dataset resulted in poorer performance. It remained difficult, however, to simplify extremely tough drawings. It performed worse than HED [31] and RCF [32], which were pretrained on ImageNet if their models were trained only on BSDS500. Xu et al. [33] found that, in simplifying a very sketchy and difficult drawing, a simplification network trained with a simple loss, such as pixel loss or discriminator loss, may fail to retain the semantically significant information. Due to various design trends, however, some artists may add auxiliary lines. The auxiliary lines during their preparation were not included. Their network cannot, however, erase these auxiliary lines as rough drawings. Secondly, when image resolution is too poor, it becomes difficult; the network eventually simplifies the diagram and loses the information. Also, the structured sketch was too simple and limited, since the sketches drawn by artists have little deviation when initial lines are taken into account. In addition, this sort of line may be inconsistent with real-world lines.

In late 2019, vectorizing line drawings is required for digital workflows of 2D animation and technical design, but it is a challenge, particularly at junctions, because of the uncertainty of topology. Existing methods of vectorization are either poorly accurate or not able to handle high-resolution images. Guo et al. [34] suggested a two-stage line drawing of vectorizing methods that examine global and local topology to deal with a range of challenges involving various kinds of complex junctions. Visually higher reconstruction precision was achieved compared to previous methods. Their approach enabled fast computing speeds to process high-resolution images. Even with only 10% Gaussian noise, their proposed LSNet cannot detect junctions. Thus, the TRNet approach struggled with incorrect junction candidates to reconstruct its topology. And its final vectorization results were greatly affected. Furthermore, their proposed approach includes no mechanism for simplifying strokes. That is why the effects of these images are fragile in their vectorization.

In 2020, there were plenty of attempts by researchers to solve these issues with rough sketches using deep learning. Exemplification is considered a central focus of deep learning and machine learning techniques that can be used more generally in geometry. Many forms of deep networks differ in terms of performance, consistency, and applicability. Smirnov et al. [35] proposed a deep learning system for predicting primitive parametric shapes. By expressing shapes as primitive collections, transformations and arbitrary resolution were easily applied while only a small representation was stored. In addition, they generated consistent parametric representations across inputs, which helped them to learn the joint contributing construction and predictable correspondences between shapes, enabled retrieval tools, exploration, transferring of style and structure, and so on. Their terminology not only extended Chamfer's distance but also resulted in robust loss functions, which enhanced the accuracy of the results of different tasks. However, the main shortcoming of their method was the need for the primitives to be close-form distances. Even for clean data, the combinatorial problem of defining the greatest succession of Boolean operations for a certain input would be especially difficult. Also, high loss outliers were normally explained by noisy information; either they were not English letters in the upper case or they had a rare structure.

A system for vectoring drawings like floor plans, geometric drawings, and 2D CAD images was introduced by Egiazarian et al. [36]. Two critical steps (initial cleaning and initial positioning of primitive images) use the neural grids that are trained in the combination of synthetic and real. Most of the time, a neural network will direct the primitives to the correct location. Its geometric precision, however, was usually insufficient. Thus, the pipeline improved with the optimization stage, which modified primitive parameters to improve the fit. Liu et al. [37] introduced a method of learning how to create 3D model line drawings. Their studies showed that their approach made considerable advances in inline drawing over modern standards when tested on standard sketch datasets, resulting in sketches that were close to those created by professional human artists. The involvement of the image interpretation module at assessment time was not considered. However, it is modified by the neural ranking module (NRM). They also tried to overcome the limitations by tuning the parameters by employing an in-depth grid search, which reduce the average Chamfer distance in the training dataset, but this led to unsatisfactory results.

Recently, Yan et al. [38] introduced the first criteria for assessing and focusing research on clean-up. Their metrics measured the similarity between automatically cleaned rough drawings and the artist's generated ground truth, the complexity, and unrest of rough drawings, and for rough sketch cleanup, they described their problem statement broadly, hoping many cleanings of the ground truth by professionals can be accepted (low ambiguity), and that a similar result can be obtained algorithmically in the future. A further “iteration” of the artwork, including inking by Simo-Serra et al. [39], specified a problem statement. There were no vaguer problem statements in their dataset. They have the original artist's refinement on two of their rough drawings.

In this paper, we propose a deep learning model based on the architecture known as the encoder-decoder network. This model is for cleaning line drawings and image pixels noise removal, as well as eliminating the unwanted background of the rough sketch images. Our model was trained on various datasets as a raster. We converted the dataset used in [23] into raster images. Other datasets are already in raster images. Our method reduces the time complexity, the time of model training, and the efficiency of cleaning rough sketch images with high accuracy.

## 3. Methodology

This section describes the proposed method of simplification for cleaning up sketched drawings using a deep learning model. The objective of this methodology is to build and automatically convert rough sketches into clean, simplified drawings. This method is capable of directly simplifying rough raster sketches with any image size.

### 3.1. Rough Sketch Dataset Preprocessing

#### 3.1.1. Data Collection

Data preprocessing is a very important step for training deep learning models. In this paper, the preprocessing is done as follows: first, collect the data, then split the data into input and target, and finally, data augmentation is applied.  Table 1 describes the datasets and the number of samples. The total number of rough drawing sketches images is 316. The size of the datasets that are publicly available is limited; so, we increased the number of samples by implementing augmentation techniques such as equalizing, adding noise, and slurring for all datasets. The results are 1260 rough drawing sketches images and 1260 cleaned up rough drawing sketches images. After that, Python was used for image renaming and resizing images to (424 × 424).

The fully connected neural networks model will train on three publicly available datasets. The data consists of the input data as rough sketch images and the target as cleanup images, as described in Table 2. From the first row of the samples from [23], we selected 181 rough drawing sketches. The second row in the samples from [40] consists of 64 rough line drawing sketches. The third row in the samples from [12] consists of 71 rough line drawing sketches.

Dataset 1 was proposed by [23] and consisted of 430 rough-drawn images. The targets of this dataset are 1675 images in SVG format. Each image as an input has four outputs, each with a different clean filter. The target image for this dataset has been converted from Scalable Vector Graphics (SVG) format into a raster image using the reaConverter Pro v7 programme to use for our model, which is based on raster images. The rough-sketch images are cleaned up by four professionals in the arts. They used Photoshop and Illustrator, and their dataset is publicly available on the internet. In the end, we get only 181 images for input and another 181 for a target.

### 3.2. Model Architecture

This subsection described in detail the model layers, the downsampling network, and the upsampling network for the cleanup of the rough sketch images. Downsampling networks and upsampling are effectively used to keep the connection information between the pixels of an image. A fully connected neural network (FCNN) is a type of deep learning network that depends on the total interconnection between all the nodes or neurons in one layer and the output connected to the nodes or neurons in the next layer. Fully connected networks have some advantages. One of the most important advantages is “structure agnostic,” which means there are no special assumptions needed to be made about the input. The layers in FCNN are a good choice for the sketch image cleanup. The FCNN model is trained by taking several sketch images as the inputs and the cleaned-up sketch labels as the outputs.

In our model, we first implement a downsampling network with FCNN and then an upsampling network. The CNN has been used in downsampling to generate abstract representations of the input sketch image. In the upsampling network, the abstract of sketch image representations is upsampled by applying various methods to make the images' spatial dimensions the same as the input image. This concept of the deep learning network is called the encoder-decoder network. Here are the details of the downsampling network and the upsampling network:

#### 3.2.1. Downsampling

In image processing, an autoencoder is a kind of neural network that copies the values of the input image to the output values of the image, as shown in Figure 3. The interesting part of the model is the hidden layers when training the model. The hidden layers consist of the number of neurons when the neurons of the hidden layers are less than the layers of input. In this case, hidden layers can be able only to extract essential values from the input image. So, the network will learn only the most common patterns of the images and ignore the “noise.” However, in an autoencoder model, the dimensions of the hidden layers must be smaller than those of the input or output layer. When the number of neurons in the hidden layers is greater than in the layers of input, the network will generate a copy of the input, including the noise, without extracting any essential information. In order to solve those cases, we proposed an autoencoder network with FCNN for the cleanup of the rough sketch images.

Instead of stacking the data, autoencoders have a convolution layer that can hold the input image spatial information the same as it is and extract the information softly.  Figure 4 shows how a flat 2D image is extracted into a thick square Conv1, then keeps going to become a long cubic Conv2 and another longer cubic Conv3. In our paper, the input image of this model is 424 × 424 = 179776 pixels. The images will pass through a number of channels, kernels, layers of convolution, and transposed convolution. We will explain that in an upcoming section. This process is designed to retain the spatial relationships in the data and is called encoding. In the middle of the architecture are fully connected layers that are composed of neurons. After that, comes the decoding process that flattens the cubes into a 2D flat image. In Figure 4, the encoder and the decoder correspond and are demonstrated.

### 3.3. FCNN model and Its Hyperparameters

There was a need to use a neural network capable of accepting input images of any size without restrictions and capable of classifying them. The first thing that we thought about was fully convolutional networks (FCCN). The idea of using a fully connected neural network came to mind. FCNN is a type of neural network without any “dense” layers; its basic structure is like the classical CNNs. In this experiment, the FCNN model encompasses 1 × 1 convolutions, which carry out the same task in fully connected layers (dense layers). The limitation of the FCNN is the number of features, which sometimes leads to overfitting. While creating the model, there are some hyperparameters that you will come across for training the network from scratch, and fine-tuning should be done to avoid the overfitting problem.

Through neural network techniques, the network structure is determined by hyperparameters, which are the different factors and variables that control the network's structure. Deep learning techniques these days are based on modified channels, kernels, and stride parameters. A hyperparameter is a training parameter set by a machine learning engineer before training the model. Model parameters are the variables that the machine learning model learns from the data while it is being trained on an existing dataset. Most of the development of the models is based on the hyperparameters, such as deep learning provides many pretraining models developed based on the concept of hyperparameters such as VGG16, VGG19, and MobilNet v2, which are used for image classification and segmentation. Based on that, our model was developed by modifying the channels and the kernels with flat layers.

We aim to introduce a few concepts before going into the training process: layers, channels, feature maps, filters, and kernels. Layers and filters are on the same level in the hierarchical structure, while channels and kernels are one level below. The terms “channels” and “feature maps” refer to the same concept. A layer can have many channels (or feature maps), for example, if the inputs are RGB images, the input layer has three channels. A layer's structure is commonly referred to as a channel. Similarly, the structure of a filter is described by the term “kernel” [41].

#### 3.3.1. Downsampling and Upsampling in the Convolutional Layer

To go deeper into how the model works, Figures 5 and 6 are used, which show the downsampling and upsampling, respectively. In the downsampling task, the input of the convolutional layer is 5 × 5, and the output after using a 3 × 3 kernel filter with 2 strides is matrix 2∗2. In up-sampling, we used transposed convolution. It works the opposite of convolution, which means reconstructing the input. In Figure 6, transposed convolution has 2 × 2 input with a 3 × 3 kernel and when strided by 2, the output will be 5 × 5, which means the matrix before convolution. Note that the image is a matrix of rows and columns, and as is known in calculating algorithms, it is done according to mathematical operations.

*(1) The Convolution Layer*. Convolutional layer is one of the main components of convolutional neural network used for features extraction [42–47]. The feature maps, or features, like the green and blue squares in Figure 5, are extracted during the convolution process. The relationship between pixels in the input image is preserved by these squares. The input of the convolutional layer is 5 × 5 and the output, after using a 3 × 3 kernel filter with 2 strides, is a matrix 2 × 2 format. Filtering refers to the method of generating the scores.

*(2) Stride*. The stride parameter indicates how many pixels across the input matrix are moved. When stride is set to 1, the filters are shifted by one pixel. When stride is set to two, the filters are shifted in two-pixel increments, and so forth. In other words, the expressiveness of the model may be boosted by substituting stride convolution for max-pooling (or any other sort of pooling). Stride convolution may be used to downsample photos. A 3 × 3 convolution with stride 2 and padding 1 converts an image of 4 × 4 pixels to 2 × 2 pixels in Figure 6.

The drawback of stride convolution is that it expands the number of parameters in the CNN model training time. Springenberg et al. [48] did great compassion between max-pooling and stride convolution. They found that stride convolution can be better for feature maps. With additional filters, the model can extract a larger number of features. More features, on the other hand, mean more training time. In this paper, to extract the features, we applied the lowest number of filters.

*(3) Padding*. One technique is used to keep the same dimension of the original sketch image by adding zeros to the boundary of the image when we define it. Otherwise, the network will drop a part of the original image.

*(4) The Rectified Linear Unit (ReLU)*. The rectified linear activation function is a piecewise linear function that outputs the value directly when the input is positive and zero when the input is negative. It is mathematically defined as *y* = max (0, *x*). As a consequence, by using ReLU, the amount of compute required to operate the neural network is prevented from rising exponentially. The computational cost of adding additional ReLUs grows linearly as the size of the FCNN increases [49].

*(5) The Conv2D in our Model*. Conv2D (filters, kernel_size, activation = ^“^relu,^”^strides = 2) is as follows: the height and width of the 2D convolution window are the kernel size. In our example, the kernel size will be (3, 3). The stride is the number of pixels in the input matrix that shift. We used flat-convolution stride 1 because the filters are used to pass on one pixel at a time on one image. In Conv2D, we use stride 2 because we move the filters 2 pixels at a time. When the kernel size is small, the stride is also small that it increases the number of the features extracted from the images. In our paper, we aim for this by varying the kernel size and stride. In addition, to keep the features of the image the same, we used padding = ^“^same^”^ to pad the picture with zeroes to fit the picture.

In the convolution downsampling, we created several convolution layers. In the downsampling phase of Figure 4, there are three layers labeled Conv1, Conv2, and Conv3. The input image with shape = (424, 424, 1) declares as the input 2D image that it is 424 by 424. Notice that Conv1 is inside of Conv2, and that Conv2 is inside of Conv3. With channels (64, 128, 256), respectively, the output from Conv1 is the input to Conv2, and the output of Conv2 is the input to Conv3. The three convolutional layers in upsampling include 5, 8, and 8 flat-convolutional layers, respectively. This means the first layer is conv1, kernel size (3 × 3), and stride 2, with 5 flat-convolution and 64 channels. The second layer is Conv2, kernel size (3 × 3), and stride 2, with 8 flat-Convs and 128 channels. The third layer is conv3, kernel size (3 × 3) and stride 2, with 8 flat-Conv and 256 channels. As illustrated in Figure 7, each layer appears as a multichannel image of size h w, where h and w are the height and width, respectively, of the image. We rely mostly on 3 × 3 convolution kernels and upsampling layers to decrease the number of parameters in the entire model. After each convolution block, we need regularization (batch-normalization). Regularization to avoid overfitting helps with quick convergence.

#### 3.3.2. Upsampling

The intermediate layers in FCCNs often get smaller (albeit often deeper) as striding reduces the height and width dimensions of the tensors, which presents a logistical challenge. To upsample the intermediate tensors to fit the width and height of the original input image, FCCNs utilize “deconvolutions” or effectively backward convolutions. In upsampling, we used transposed convolution. It works opposite to the convolution, which means to reconstruct the input.

*(1) Conv2DTranspose*. Transposed convolutions are more flexible and have more complex implementation than the classical nearest neighbor or bilinear upsampling methods. These layers are used to apply some learnable parameters to up-sample the input feature map to a desired output feature map. It is necessary to indicate the number of filters as well as the size of each filter's kernel. One of the main considerations in this layer is stride. In a typical convolutional layer, stride or strides refers to the application of a filter scanning across an input, resulting in a smaller output. However, in transposed convolutions from a distribution perspective, stride scans over the output, which increases the size of the output. Because stride over the output is equal to a fractional stride over the input, it is also known as fractionally stride convolution. A stride of 2 can pass over the output. This, for example, equals 1/2 stride over the input. Strides are responsible for the upscaling effect of transposed convolutions. The Conv2DTranspose layer takes images as input and delivers the operation's outcome.

The Conv2DTranspose performs both an upsample and a convolution. The Conv2DTranspose both upsamples and performs a convolution. Because the upsampling process is performed by the stride behavior of the convolution on the input, we must provide the number of filters and their sizes, just as we do with Conv2D layers and stride size. In Figure 8, transposed convolution has a 2 × 2 input with a 3 × 3 kernel, and when strided by 2, the output will be 5 × 5, which means the matrix before convolution.

The height and width of the input will be reduced after applying a convolution block to it, based on the strides and kernel size. It is possible that the following convolution block may not work properly if the input image is too small (which must be greater than or equal to the kernel size).

*(2) The Algorithm Steps of Upsampling*.

1. Determine how many convolution blocks you will be stacking
2. Stack the convolution blocks with increasing numbers of channels on any input shape, such as (128, 128, 3)
3. To make the model, you will need to first build it. Use the summary() function to see the final shape of each layer
4. Verify the final convolution block's output dimensions which are (1, 1, number of filters) (this will be input to a fully connected layer).
5. To meet the criteria in step 4, experiment with different input shapes, kernel sizes, and strides. What you need is the smallest possible input shape, along with other configurations, to satisfy your network's requirements

Those steps are based on a trial-and-error approach to finding the smallest input dimension. Because they mirror the functionality of the FC layer along with the number of filters dimension, the input dimension to the 1 × 1 convolution might be (1, 1, num of filters) or (height, width, number of filters). After the 1 × 1 convolutions, the input to the last layer (the sigmoid activation layer) must be of a fixed length.

*(3) The Transposed Convolution in our Model*. Transposed convolution (also known as deconvolution or fractionally stride convolution) is an approach for upsampling an image with parameters that can be learned. Transposed convolution, on the other hand, is the opposite of typical convolution in that the input volume is a low-resolution image, and the output volume is a high-resolution image. The transposed convolution repeats the rows and columns of the data by size [row_number] and size [columns_number], respectively. So, we start the first Conv2DTranspose with the number of filters (128), and the kernel size is (3 × 3) and stride by 2. The stride is the number of pixels in the input matrix that shift. We used Transposed Convolution Stride 2 because we shifted the filters 1 pixel at a time. The stride is very important. It is key to getting the high-resolution image as an output. They are also Conv2DTranspose 2 and Conv2DTranspose 3 with the number of filters (64 and 32), the kernel size of (3 × 3), and stride by 2. Each layer gets input from the previous layer.  Figure 9 shows the steps of passing the image from Conv2DTranspose 1 to Conv2DTranspose 2 and then Conv2DTranspose 3. In each step, the size is increased. Finally, we get the output image as the original, with the unwanted pixels removed.

## 4. Experimental Results and Discussion

This section discusses the results obtained from this experiment. The FCNN model was trained on three datasets combined from three standard datasets. The first dataset proposed in [23] was published in 2020, and the target is in Scalable Vector Graphics (SVG) format. Our paper is the first one that used this dataset and converted it to a raster format, as well as using other two raster image datasets. The dataset evaluated in our experiment consists of 1260 rough sketch images as input and 1260 clean images as a target. We reduce the number of parameters in the full model by relying primarily on 3 convolution kernels and the upsampling layers, which use 3 × 3 kernels. In this model, the 3 convolution downsampling layers are followed by flat layers, and the 3 convolution upsampling layers are followed by flat layers. The flat layers which follow the convolution downsampling are 5, 8, and 8, respectively, and in upsampling, they are 8, 5, and 5, respectively. In our model, we increased the number of convolutional and flat layers to extract the maximum number of features from the input image, which led to a good accuracy result. We built our model using the most popular deep learning library, TensorFlow, which is supported by the Python language. The model was trained for 300 iterations with a batch size of 6, which took roughly 12 hours on a Core i7 laptop with an 8 GPU.

### 4.1. Performance Measurement

Mean square error (MSE) pooling is a pooling operation that calculates the square mean for patches of a feature map and uses it to create a downsampled (pooled) feature map in (2). It is usually used after a convolutional layer. In our model, the loss of the model is decreased by an increase in the epochs, as shown in Figure 10.

(2) $$\begin{array}{c} \text{MSE}=\frac{1}{N}\overset{N}{\underset{i=1}{\sum }}{\left(f_{i}-y_{i}\right)}^{2}, \end{array}$$

where *N* is the number data features, *f*_*i*_ is the value of pixel returned by the model, and *y*_*i*_ is the actual value of pixel *i*.

Training the model with 6 batch sizes and 300 epochs, the model achieves a minimum error rate of 0.08, which is shown in the root mean square (RMS) of the running is 0.08. The model takes around 12 hours of training. The training accuracy result is shown in Figure 11, which reaches around 970~98%.

### 4.2. Comparison with the Existing Methods

In comparison, we tested our model with the same datasets employed in previous works and got the same result for the same images, that they used. Then, we used their images from their research papers to test our model. The training of the model depends on a set of hand-drawn images as input, in contrast to the image of the target that is being trained to build a knowledge base that will be used to clean and improve the images during implementation in real-time testing. We proposed a deep learning model that takes rough sketch images (pencil and scanned images) and generates simplified, stylized vector data. This topology is optimized to drive the final vectorization method to transform the input bitmap into a high-quality raster image by removing open curves. Techniques based on convolutional neural networks are used in Mastering Sketching [12] and Real-Time Inking [39].  Table 3 shows our comparative model for cleanup rough sketch images with state-of-the-art methods. The two algorithms use different resolution dependences to combine multiple rough strokes. When high image size is used for simplification and clean-up tasks, the Mastering Sketching approach fails. Fidelity vs. simplicity [9] performed poorly in the presence of gaps in sketch images. This method cannot close the gaps in sketch images, and then the output drastically improves. The Delaunay triangulation [50] method is highly dependent on the parameters that are used in the computations. Finding a single set of parameters that works for all sketches is a difficult task. The topology-driven [7] and polyvector [10] approaches focus on faithful vectorization and do not group repeated messy strokes. Compared to the existing methods, our FCCN model is suited for sketch image clean-up with low messiness and provides higher accuracy for sketch clean-up compared to the existing methods. Our limitation is that the datasets for the cleaning up rough sketch images are not available, and there are only small dataset samples. Also, traditional methods that are used for cleanup sketch images are few. In particular, when we compare our model with the Simo-Serra et al. [11] model Table 4, their model was trained with 600,000 iterations and a batch size of 6. It takes roughly three weeks using an Nvidia TITAN X GPU. Our model is trained with 300 iterations with a batch size of 6, which takes roughly 12 hours using a Core i7 laptop with an 8 GPU.

Real-time testing is the process of testing deep learning models that operate in real time. The real-time testing is carried out in order to find and assist in the correction of problems in deep learning models. In testing, it is important to ensure that the program is not only error-free but also that it offers the user with the functionality that they demand. With that in mind, we randomly selected two sketches from the internet that are not in our dataset to test the capability of our model and how functional and reliable it is. As it can be seen from Table 5, the two sketches on the left are the inputs, which are shady and unclear, while the sketches on the right are the outputs produced by our model, which vividly illustrates all the details of the sketch with higher resolution and clarity.

## 5. Conclusion

This paper presents a deep learning-based model that automatically converts rough raster sketches images into high-quality simplified images. The proposed model is built on multilayer convolutional processes to provide promising results, and it can handle very complicated pencil and scanned images, which can be collected from different sources. Additionally, our proposed stacked convolutional structure is suitable for simplifying the curves and strokes in such images and can handle sketch images of any size. We also introduce a new dataset neatly prepared for an implementation task of our model to be trained and tested to simplify sketch images. The results of the experiments showed that our model outperformed the state of the art in sketch image simplification, providing better results and a lower computation time compared to the existing methods. The obtained results clearly showed that hyperparameter optimizations led to better performance of the proposed model. We believe that our proposed method is a significant step in the integration of sketch simplification into the daily workflow of designers and artists.

## Figures and Tables

**Figure 1:** Inputs and outputs of our testing result for sketch images.

**Figure 2:** (a) A tangent field used by Chen et al. [18] cannot capture a collection of directions present at a junction point. (b) Bessmeltsev et al.'s frame field on a similar input is a natural representation of the directions at a junction. Input image from Bessmeltsev et al. [10].

**Figure 3:** Demonstration of the Down-sampling, flat-convolution, and up-sampling.

**Figure 4:** The model architecture.

**Figure 5:** Demonstration of the convolution.

**Figure 6:** Demonstration of the stride convolution [11].

**Figure 7:** Illustration of the channel and kernel.

**Figure 8:** Demonstration of the transposed convolution.

**Figure 9:** Demonstration of the transposed convolution of the three layers.

**Figure 10:** The training loss of the model.

**Figure 11:** The training accuracy of the model.

**Table 1:** Described the datasets and the number of the samples.

Dataset 1 [23]	Dataset 2 [40]	Dataset 3 [12]	Total rough drawing sketches images (input)	Total cleanup rough drawing sketches images (target)	The images after augmentation (input)	The images after augmentation (target)
181 rough drawing sketches images	64rough drawing sketches images	71 rough drawing sketches	316	316	1260	1260

**Table 2:** Shows the samples of the datasets.

Rough input image			
Target image			

**Table 3:** Comparisons with the Simo-Serra et al. [11] model and Liu et al. [51] model.

Rough sketch image (original)	Ground truth [38]	Our FCNN model	Mastering Sketching [12]	Real-Time Inking [39]	Polyvector [10]→ stroke aggregator [23]	Topology-driven [7]	Topology-driven [7]→stroke aggregator [23]	Delaunay triangulation [50]	Fidelity simplicity [9]
									
Rough sketch image (original)	Ground truth [38]	Our FCNN model	Mastering Sketching [12]	Fidelity simplicity [9]	Topology-driven [7]	Polyvector [10]	Polyvector [10]→ stroke aggregator [23]	Delaunay triangulation [50]	Topology-driven [7]→ Stroke aggregator [23]
									
Rough sketch image (original)	Ground truth [38]	Our FCNN model	Mastering Sketching [12]	Real-Time Inking [39]	Polyvector [10]	Topology-driven [7]	Stroke aggregator [23]	Polyvector [10]→ Stroke Aggregator [23]	Fidelity simplicity [9]
									

**Table 4:** Comparisons for cleanup rough sketch images with state-of-the-art methods.

	Input image	Cleanup using our model after 300 iterations	Simo-Serra et al. [11]	Liu et al. [51]
(a) Fairy				
(b) Mouse				
(c) Car				

**Table 5:** More results are produced by our model.

Input rough sketch images	Output clean up images
	
	

## Data Availability

Dataset 1: https://www.cs.ubc.ca/labs/imager/tr/2018/StrokeAggregator/. Dataset 2: https://www.arxiv-vanity.com/papers/1603.07285/. Dataset 3: https://esslab.jp/~ess/en/research/sketch_master/.
